RETRACTED

# Alpha-ketoglutarate promotes skeletal muscle hypertrophy and protein synthesis through Akt/mTOR signaling pathways

**DOI:** 10.1038/srep26802

**Published:** 2016-05-26

**Authors:** Xingcai Cai, Canjun Zhu, Yaqiong Xu, Yuanyuan Jing, Yexian Yuan, Lina Wang, Songbo Wang, Xiaotong Zhu, Ping Gao, Yongliang Zhang, Qingyan Jiang, Gang Shu

**Affiliations:** 1 National Engineering Research Center for Breeding Swine Industry, College of Animal Science, South China Agricultural University, Guangzhou, Guangdong, 510642, China; 2 ALLTECH-SCAU Animal Nutrition Control Research Alliance, South China Agricultural University, Guangzhou 510642, PR China

## Abstract

Skeletal muscle weight loss is accompanied by small fiber size and low protein content. Alpha-ketoglutarate (AKG) participates in protein and nitrogen metabolism. The effect of AKG on skeletal muscle hypertrophy has not yet been tested, and its underlying mechanism is yet to be determined. In this study, we demonstrated that AKG (2%) increased the gastrocnemius muscle weight and fiber diameter in mice. Our *in vitro* study also confirmed that AKG dose increased protein synthesis in C2C12 myotubes, which could be effectively blocked by the antagonists of Akt and mTOR. The effects of AKG on skeletal muscle protein synthesis were independent of glutamate, its metabolite. We tested the expression of GPR91 and GPR99. The result demonstrated that C2C12 cells expressed GPR91, which could be upregulated by AKG. GPR91 knockdown abolished the effect of AKG on protein synthesis but failed to inhibit protein degradation. These findings demonstrated that AKG promoted skeletal muscle hypertrophy via Akt/mTOR signaling pathway. In addition, GPR91 might be partially attributed to AKG-induced skeletal muscle protein synthesis.

Skeletal muscle, which is the most abundant tissue in the body of mammals, has a wide variety of important functions^1^. Skeletal muscle mass is determined by the dynamic balance between protein synthesis and degradation^2^,^3^. The protein synthesis of skeletal muscle has been proven to be affected by different nutritional and physiological factors, such as amino acids^4^,^5^, glucose^6^, exercise^7^, insulin-like growth factor-1 (IGF-I), and insulin^8^. Notably, the mammalian target of rapamycin (mTOR) plays a critical role in promoting the protein synthesis of skeletal muscle^9^, which is mediated by its downstream P70S6K1, S6, and 4E-BP1^10^,^11^,^12^,^13^. The activation of forkhead box O (FoxO) transcriptional protein family members FoxO1 and FoxO3a induce the degradation of protein by increasing the expression of MuRF1 and MAFbx^14^,^15^.

Alpha-ketoglutarate (AKG) is a crucial intermediate in the tricarboxylic acid (TCA) cycle and is also a product of glutamine deamination (glutaminolysis)^16^,^17^,^18^. The mTOR directly senses the intracellular content of key amino acids, such as glutamine and leucine, in potentiate protein synthesis^19^. However, limited studies have been conducted on the role of AKG in skeletal muscle hypertrophy. Yao *et al*. reported AKG-enhanced protein synthesis in intestinal porcine epithelial cells^20^. AKG was believed to mediate the function of amino acid in active mTOR in Hela cells^16^. These findings led to the hypothesis that AKG might benefit skeletal muscle protein synthesis and promote muscle hypertrophy.

RETRACTED

Two membrane proteins, namely, the G protein-coupled receptors (GPR) 91 and GPR99, were identified to sense some intermediates in tricarboxylic acid and mediate the adaptation of different energy metabolism statuses^21^. GPR99 was considered a typical receptor for AKG^22^, whereas GPR91 responded to succinate^23^,^24^. Given that AKG is a dicarboxylic acid similar to succinate, GPR91 and GPR99 could sense extracellular AKG concentration^21^. However, whether GPR91/99 is required for AKG modulated skeletal muscle protein synthesis has not yet been tested.

Thus, the main purpose of this paper is to explore the role of AKG in regulating protein synthesis in skeletal muscle and to determine a potential signaling pathway. AKG could dose-dependently induce skeletal muscle hypertrophy and enhance protein synthesis via the Akt/mTOR signaling pathway. Our observation indicates that GPR91 is involved in AKG-facilitated protein synthesis. However, we should emphasize that the effects of AKG on skeletal muscle protein synthesis were independent of glutamate. Our results represent the first identification of AKG in promoting skeletal muscle hypertrophy and highlight the bioactive and nutritional value of ketonic acids.

## Results

### AKG-promoted skeletal muscle hypertrophy in C57BL6/J mice

To test the effect of AKG on skeletal muscle hypertrophy, C57BL6/J mice were treated with 1% and 2% AKG via drinking water. Compared with the control, serum AKG level was largely elevated in the 2% AKG group (Fig. 1a); this group also had higher daily body weight gain than the control group (Fig. 1b). In addition, 2% AKG administration reduced the abdominal fat of mice and enhanced the gastrocnemius muscle weight (Fig. 1c) and fiber size (Fig. 1d) of mice compared with the control. The liver index remained unchanged. Notably, the expression of two protein degradation genes, 4E-BP1 and MAFbx, in gastrocnemius tissue were significantly reduced (Fig. 1e,f). By contrast, the phosphorylation of Akt, mTOR, and S6 increased (Fig. 1f) after 2% AKG treatment. Immunocytochemistry (IHC) data illustrated the AKG-enhanced phosphor-S6 levels in gastrocnemius tissue (Fig. 1g). These findings suggest that AKG promotes skeletal muscle hypertrophy, which is probably caused by enhanced protein synthesis and reduced protein degradation.

RETRACTED

### AKG increased the protein synthesis of C2C12 myotubes

As expected, our further *in vitro* study also confirmed that AKG (0.5 and 2 mM) could dose-dependently increase cellular protein levels and the puromycin incorporation of C2C12 myotubes (Fig. 2a,b). In addition, both 0.5 and 2 mM AKG could significantly increase the expression of MyHC and promote the phosphorylation of mTOR, S6, 4E-BP1, and eIF4E while inhibiting that of eIF2^α^ (Fig. 2c). IHC data also displayed that both the MHCII and the phosphorylation of S6 positive myotubes were clearly increased when exposed to AKG (Fig. 2d). These results support the hypothesis that AKG promotes protein translation and synthesis in C2C12 myotubes.

### Effects of AKG on protein synthesis were not mediated by its metabolite

Glutamate is the main metabolite of AKG. To determine whether glutamate is required for AKG-induced protein synthesis, C2C12 myotubes were exposed to AKG or glutamate. Consistent with early observation, AKG increased cellular protein synthesis (Fig. 3a) and the phosphorylation level of mTOR, S6, and 4E-BP-1 but decreased the level of eIF2α (Fig. 3b,c). However, glutamate did not affect the protein synthesis of C2C12 myotubes and S6 *et al*. These findings indicate that AKG has a direct effect on protein synthesis, which is independent from its metabolite.

### AKG promoted C2C12 cells protein synthesis through mTOR signaling pathway

The mTOR signaling pathway is crucial for protein synthesis. In this study, we observed that the phosphorylation level of mTOR, P70S6K1, S6, 4E-BP1, and eIF4E increased in C2C12 myotubes when exposed to 2 mM AKG for 1, 2, and 4 h (Fig. 4a). To test whether mTOR pathway is involved in-AKG induced protein synthesis, C2C12 myotubes were co-treated with AKG and the specific inhibitor of mTOR (rapamycin). Results showed that rapamycin potently abolished the effects of AKG on cellular protein content (Fig. 4b), protein synthesis (Fig. 4c), and phosphorylation of mTOR, S6, and 4E-BP1 (Fig. 4d). These data suggest the essential role of the mTOR signaling pathway in AKG-induced C2C12 cells protein synthesis.

### Akt-mediated AKG in active mTOR signaling pathway

The mTOR integrates diverse hormones and energy status signals via PI3K/Akt^25^,^26^ or directly senses intracellular amino acids concentration^27^. To determine whether Akt mediates AKG actions on mTOR activation, C2C12 myotubes were subjected to AKG alone or co-treated with PI3K/Akt inhibitor (LY294002). Notably, the phosphorylation of Akt, FoxO1, and FoxO3a was significantly increased by AKG at 1, 2, and 4 h. Similarly, the protein level of 2 FoxO downstream protein, namely, MuRF1 and MAFbx, also decreased (Fig. 5a). The effects of AKG on protein synthesis (Fig. 5b), Akt/FoxO1 (Fig. 5c), and mTOR/S6 (Fig. 5d) were effectively blocked by LY294002. These observations demonstrate that Akt is involved in AKG-induced mTOR activation and protein deposition.

RETRACTED

### The role of GPR91 and GPR99 in AKG-induced protein deposition of C2C12 cells

GPR91 and GPR99 senses the intermediate in the tricarboxylic acid cycle^21^. We first checked the mRNA expression of these two receptors in C2C12 myotubes and found that GPR99 mRNA is too minimal to be detected (Fig. 6a). By contrast, C2C12 myotubes highly expressed GPR91 (Fig. 6a), which could be further up-regulated by AKG (Fig. 6b). This observation raises the possibility that GPR91 might be involved in AKG-induced protein synthesis. To determine whether GPR91 mediated the role of AKG in protein deposition, C2C12 myoblasts were transferred with GPR91 siRNA to knock down its gene expression. The effect of AKG on protein deposition was partially attenuated by GPR91 knockdown (Fig. 6c). Moreover, the activation of mTOR and S6 and the inactivation of 4E-BP1 by AKG disappeared in GPR91 knockdown cells (Fig. 6d). By contrast, GPR91 knockdown failed to abolish the effects of AKG on the mRNA expression of MuRF1 and MAFbx (Fig. 6e). This paradoxical evidence suggests that GPR91 might be involved in the AKG-induced increase of protein synthesis but not in the inhibition of protein degradation.

### AKG enhanced protein synthesis in the skeletal muscle of mice

To further verify the effects of AKG on protein synthesis in skeletal muscle, mice were injected with 0.6 g/kg AKG for 1h and 3 h, respectively. Although the differences is not statistically significant, we also find AKG had a tendency to increase the protein synthesis (puromycin incorporation, *P* = 0.058) (Fig. 7a) and increased the expression of MyHC but decreased that of MuRF1 and MAFbx in gastrocnemius muscle (Fig. 7d). Similarly, we observed that AKG activated S6 and eIF2^α^, and inactivated FoxO1 and 4E-BP1 in the gastrocnemius muscle (Fig. 7b,c). Further, the phosphorylation levels of Akt and mTOR were significantly elevated 1 h after AKG injection (Fig. 7e), which disappeared 3 h after injection (Fig. 7b,c).

## Discussion

In this study, we first identified the novel role of AKG in skeletal muscle hypertrophy. Skeletal muscle is the largest plastic organ in the body^28^,^29^. The size of skeletal muscle fiber is influenced by different physiological status, such as mechanical stress^30^, physical activity^31^, availability of nutrients, and growth factors^32^. Excessive loss of muscle mass is associated with an imbalance between protein synthesis and protein degradation^33^,^34^. Nutritional therapy is one of the most convenient and effective methods to increase skeletal muscle mass. Thus, our results suggest that the oral administration of AKG significantly increased the weight of gastrocnemius muscle in C57BL6/J mice, which was attributed to a large fiber size.

RETRACTED

Generally, muscle hypertrophy is related to high protein synthesis and low protein degradation. As an enriched α-keto acids, AKG is involved in the nitrogen and protein metabolism of humans and other animals^35^. Ornithine AKG-reduced nitrogen losses in rats fed on a nitrogen-free diet have been reported^36^. Some clinical data also demonstrated AKG-preserved protein synthesis and free glutamine after surgery^37^. Moreover, 2 mM AKG increased protein synthesis by 50% in IPEC-J2 cells^20^. We further identified the novel role of AKG in skeletal muscle hypertrophy. S6 and 4E-BP1 are two mTOR downstream signaling moleculars that play key roles in protein synthesis^38^,^39^. Thus, the increased phosphorylation level of S6 and 4E-BP1 indicates the acceleration of protein translation. These results indicated that AKG promoted the protein synthesis of skeletal muscle.

Identifying the underlying mechanism of a nutrient is a complicated process because most of nutrients are metabolized to their subsequent metabolites. The same is true for AKG, which generates glutamate by glutamate synthase^9^,^40^. The present study showed that AKG significantly increased the MHCII expression and protein synthesis of C2C12 myotubes. Accordingly, the phosphorylation of mTOR, S6, 4E-BP1, and eIF4E was increased by AKG treatment. However, glutamate could not mimic the effects of AKG in the protein synthesis of C2C12 myotubes. Previous evidence suggests that glutamate plays a key function in nitrogen assimilation, amino acid biosynthesis, and cofactor production^41^. Moreover, glutamate reportedly enhances mucosal protein synthesis^42^. These data suggested that AKG could directly increase protein synthesis, which is independent of glutamate, its metabolite.

The fiber size of skeletal muscle is regulated in coordination by several signaling pathways, such as AMPK^43^, Akt/mTOR/FoxO^44^,^45^, Smad^46^, and IKK/NFκB^47^,^48^. Notably, the Akt/mTOR/FoxO signaling pathway is crucial in protein turnover and muscle hypertrophy^12^. On the one hand, Akt promotes the protein synthesis of skeletal muscle by activating Akt/mTOR and downstream signaling molecules S6 and inactivating 4E-BP1^49^. On the other hand, Akt increases the phosphorylation of FoxO1 and FoxO3a (inactivation), and therefore decreases the expression of two protein degradation-associated protein, namely, MuRF1 and MAFbx^50^,^51^,^52^. Previous studies reported that AKG increased the phosphorylation level of Akt and its downstream molecule to improve cell fate in HEK293 cells during metabolic stress^53^. In the present study, we demonstrated that AKG activated the Akt/mTOR pathway and inactivated the FoxO pathway in C2C12 myotubes. Both the Akt inhibitor (LY294002) and mTOR inhibitor (rapamycin) reversed the effect of AKG on protein deposition in C2C12 myotubes. These findings indicate that AKG increased the protein deposition of skeletal muscle via the Akt/mTOR signaling pathway.

RETRACTED

GPR91 and GPR99 sense the intermediates in the tricarboxylic acid cycle. Recently, a study considered GPR99 as a typical receptor for AKG^22^,^54^,^55^, which led to the hypothesis that AKG-induced skeletal hypertrophy might be mediated by GPR99. However, the mRNA expression of GPR99 is too minimal to be detected by qPCR, which is consistent with previous reports^23^. Unexpectedly, GPR91 is highly expressed in C2C12 myotubes. In addition, the gene expression of GPR91 was up-regulated by AKG treatment. GPR91 activation couples to a Gi/Go pathway. Nevertheless, AKG weakly inhibited the forskolin-stimulated cAMP production in 293-hGPR91 cells^21^; this finding suggests that GPR91 could sense extracellular AKG. Our data demonstrated that GPR91 knockdown partially attenuated AKG-induced protein synthesis. Therefore, future studies should further identify the receptor that mediates the effect of AKG on skeletal muscle hypertrophy.

In summary, AKG promotes skeletal muscle protein synthesis and inhibits the degradation mediated by the Akt/mTOR pathway. GPR91 might be partially attributed to AKG-induced skeletal muscle protein synthesis. These data suggest the promising application of AKG in maintaining protein turnover balance in skeletal muscle and treating muscle atrophy.

## Materials and Methods

### Animals

All experimental protocols and methods were approved by the College of Animal Science, South China Agricultural University. All experiments were conducted in accordance with “The Instructive Notions with Respect to Caring for Laboratory Animals” issued by the Ministry of Science and Technology of the People’s Republic of China. C57BL6/J mice were purchased from the Animal Experiment Center of Guangdong Province [permission number: SYXK (Yue) 2014-0136]. The mice were left to acclimate 1 week before the experimental period and maintained under constant light for 12 h and a 12 h dark cycle at a temperature of 23 °C ± 3 °C and relative humidity of 70%±10% throughout the experimental period. The mice were given access to standard pellets (crude protein 18%, crude fat 4%, and crude ash 8%). In the chronic experiment, 30 5-week-old mice were randomly divided into three groups (n = 10). Different concentrations of AKG (0%, 1%, and 2%) were supplemented by drinking water for 9 weeks. Body weight was checked weekly. At the end of the experiment, all mice were sacrificed to analyze their body composition and to collect blood samples and gastrocnemius tissue for further testing. In the acute experiment, 40 3-week-old mice were divided into four groups (n = 10) and injected by intraperitoneal with saline and 0.6 g/kg of AKG (Sigma) for 1 and 3 h, respectively. The animals were sacrificed 1 and 3 h post injection to collect gastrocnemius samples. The samples were stored at −80 °C for further qPCR and Western blot analysis.

RETRACTED

### Cell culture

Murine skeletal muscle cell line C2C12 was cultured in high glucose DMEM (GIBCO, Grand Island, NY, USA), supplemented with 10% fetal bovine serum (FBS; GIBCO), 100000 units/L of penicillin sodium, and 100 mg/L of streptomycin sulfate (GIBCO) at 37 °C in a humidified atmosphere that contained 5% CO_2_. The C2C12 myoblasts were induced differently to myotubes by a medium that contained high glucose DMEM and 2% horse serum (HS; GIBCO) for 6 days.

### Akt/mTOR pathway inhibition

To identify the underlying mechanisms of AKG on protein synthesis, C2C12 myotubes were co-treated with AKG with the Akt inhibitor 5μM LY29004 (Beyotime Biotechnology, China) and mTOR inhibitor 1 μM rapamycin (Sigma, Shanghai, China). The protein synthesis and their downstream protein levels were analyzed.

### GPR91 siRNA transfection

To knock down the expression of GPR91, siRNA of GPR91 was purchased from GenePharma Co., Ltd. (Shanghai, China) and transfected with lipofectamine (Invitrogen, Carlsbad, CA, USA) in accordance with the manufacturer’s instructions. The siRNA sequences of GPR91 were as follows: (sense) 5′-GCUCUUGCUCACUGUCAUUTT-3′; (resense) 5′-AAUGACAGUGAGCAAGAGCTT-3′; Negative control: (sense) 5′-UUCUCCGAACGUGUCACGUTT-3′; (resense) 5′-ACGUGACACGUUCGGAGAATT-3′.

### Total protein content

C2C12 myotubes were treated with 0.5 and 2 mM AKG for 48 h. Cells were washed twice with cold PBS and lysed using 200 μL radio immunoprecipitation assay (RIPA) lysis buffer that contained 1 mM PMSF and protein phosphatase inhibitor complex (Biosino Bio-Technology and Science Inc., Beijing, China). The total protein of the cell lysate was detected using a commercial kit (Thermo Scientific Technologies, Wilmington, DE, USA) and normalized by DNA content.

RETRACTED

### Puromycin assay

SUnSET method was used to measure protein synthesis *in vitro* and *in vivo* as previously described 56. For the *in vitro* study, 10 μg/ mL puromycin was added to the medium 1 h before C2C12 was collected. For the *in vivo* study, 100 μg/ mL puromycin was injected 1 h before muscle tissue collection. The incorporation of puromycin in the total protein was analyzed by Western blot.

### Western blot assay

Cells were lysed in RIPA lysis buffer that contained 1 mM PMSF. Total protein concentration was determined using BCA protein assays. After separation on 10% sodium dodecyl sulfate (SDS)–polyacrylamide gel electrophoresis gels, the proteins were transferred to polyvinylidene fluoride (PVDF) membranes and then blocked with 5% (wt/vol) non-fat dry milk in Tris-buffered saline that contained Tween 20 for 2 h at room temperature. The PVDF membranes were then incubated with the indicated antibodies, including rabbit anti-β-actin (Bioss) and mouse puromycin antibody 12D10 (Millipore); or rabbit anti-phospho-mTOR (Ser2481) and mTOR, rabbit anti-phosphor-P70S6K (Thr389) and P70S6K1, rabbit anti-phospho-S6 (Ser235/236) and S6, rabbit anti-phospho-4E-BP1 (Thr37/46) and 4E-BP1, rabbit anti-Akt, rabbit anti-phospho-Akt (Ser473), rabbit anti-phospho-Akt (Thr308;), rabbit anti-eIF4E, rabbit anti-phospho-eIF4E (Ser209), rabbit anti-eIF2α, rabbit anti-phospho-eIF2α (Ser251), rabbit anti-FoxO1, and rabbit anti-phospho-FoxO1 (Ser256) (Cell Signaling Technology, Beverly, MA, USA). The primary antibodies were incubated at 4 °C overnight and followed by the incubations of the appropriate secondary antibody (Bioss) for 1 h at room temperature. Protein expression was measured using a FluorChem M Fluorescent Imaging System (ProteinSimple, Santa Clara, CA, USA) and normalized to β-actin expression.

### RNA extraction, reverse transcript, and qPCR

Total RNAs were extracted from C2C12 myotubes and mouse gastrocnemius using TRIzol reagent (Invitrogen, Carlsbad, CA, USA) according to the manufacturer’s instructions. After treatment with DNase I (Takara Bio Inc., Shiga, Japan), total RNA (2 μg) was reverse-transcribed to cDNA in a final 20 μL using M-MLV Reverse Transcriptase (Promega, Madison, WI, USA) and random 9 primer (Takara Bio Inc., Shiga, Japan) according to the manufacturer’s instructions. β-actin was used as a candidate housekeeping gene. SYBR Green Real-time PCR Master Mix reagents (Toyobo Co., Ltd., Osaka, Japan) and sense and antisense primers (200 nM for each gene) were used for real-time quantitative polymerase chain reaction (PCR). PCR reactions were performed in an Mx3005p instrument (Stratagene, La Jolla, CA, USA). Some of the primer sequences are presented in Table 1.

RETRACTED

### Immunohistochemistry and immunocytochemistry

C57BL6/J mice gastrocnemius was sliced to 10 μm by using a frozen slicer (LEICA CM 1850, Germany). The sections and C2C12 cells were rinsed 3 times in PBS and washed in 0.3% H_2_O_2_ for 30 min then blocked for 1 h at room temperature. Subsequently, the sections were incubated in rabbit anti-phospho-S6 (Ser235/236;) overnight at room temperature. The sections were rinsed 3 times by PBS and incubated in ABC (Vector Laboratories, PK-4000) for 1 h. DAB (Sigma) was used for indirect immunoperoxidase staining. Upright microscopes were used to take photographs. Image-Pro Plus software was used for quantifying grayscale. Up to six fields of view were captured from the same location within each gastrocnemius muscle. 600 myofibres were measured per muscle. C2C12 cells were incubated overnight in rabbit anti-phospho-S6 (Ser235/236; CST) and mouse anti-MHCII (abcam) at 4 °C. The next day, the sections were transferred to biotin second antibody (bioworld) for 1 h, and the C2C12 cells were incubated in FITC second antibody (bioss). C2C12 cells were then observed and the fluorescences were quantified using Nikon Eclipse Ti-s microscopy with Nis-Elements BR software (Nikon Instruments, Japan). Up to six fields of view were captured from every groups.

### Hematoxylin-Eosin staining

C57BL6/J mice gastrocnemius was sliced to 10 μm by using a frozen slicer. Cross-sections were fixed in 4% formaldehyde at room temperature for 20 min and stained with hematoxylin and eosin^57^. The myofibres area was quantified using Image-Pro Plus software analysis. Up to six fields of view were captured from the same location within each gastrocnemius muscle. 600 myofibres were measured per muscle.

### Statistical analysis

All data are expressed as means ± standard error of the mean (SEM). Significant differences between the control and the treated group were determined by Student’s t test. One-way analysis of variance was used to test the dosage effect of AKG on protein synthesis (SPSS 18.0, Chicago, IL, USA). *P* < 0.05 represented significant differences.

## Additional Information

**How to cite this article**: Cai, X. *et al*. Alpha-ketoglutarate promotes skeletal muscle hypertrophy and protein synthesis through Akt/mTOR signaling pathways. *Sci. Rep*. **6**, 26802; doi: 10.1038/srep26802 (2016).

## Figures and Tables

**Figure 1:** Effects of α-ketoglutarate on skeletal muscle weight and fiber size in C57 BL mice. Thirty 5-week-old mice were randomly divided into three groups (n = 10). Different concentrations of AKG (0%, 1% and 2%) were supplemented via drinking water for 9 weeks. (**a**) Serum AKG level examined by AKG assay kit. (**b**) Mice daily body weight gain. (**c**) Liver index, abdominal fat index, and gastrocnemius index. (**d**) Representative images of gastrocnemius muscle stained by H&E and gastrocnemius muscle fiber area distribution. The place of arrows direction represented muscle fiber. (**e**) Relative mRNA expression detected by qPCR. (**f**) Phosphorylation levels of Akt mTOR, S6, 4E-BP1, FoxO1, and the expression of MAFbx by Western blot. (**g**) The phospho-S6 protein expression examined by IHC in the gastrocnemius of mice. The place of arrows direction represented the expression of phospho-S6. Data are presented as mean ± SEM. Different superscripts “a”/“b”/“c” represent significant differences between groups (*P *< 0.05), and *means *P* < 0.05 compared with the control. β-actin served as a housekeeping gene.

RETRACTED

**Figure 2:** AKG increased protein synthesis in C2C12 myotubes. C2C12 cells were cultured for 6 d in a differentiation medium. C2C12 myotubes were then exposed to different concentrations of AKG (0, 0.5, and 2 mM) for 48 h. (**a**) Total protein levels. (**b**) Puromycin levels detected in C2C12 myotubes by Western blot. (**c**) The phosphorylation levels of mTOR, S6, 4E-BP1, eIF4E, eIF2a, and MyHC by Western blot. (**d**) IHC analysis for MHCII and phospho-S6 in C2C12 myotubes. Data are presented as mean±S.E.M. Different superscripts “a”/“b”/“c” represent significant differences between groups (*P* < 0.05), and * means *P* < 0.05 compared with the control. β-actin served as a housekeeping gene.

**Figure 3:** Glutamate failed to promote protein synthesis in C2C12 myotubes. C2C12 cells were cultured for 6 d in a differentiation medium. C2C12 myotubes were then exposed to glutamate (2 mM) and AKG (2 mM) for 48 h. (**a**) Total protein levels. (**b**) The phosphorylation level of mTOR, S6, 4E-BP1, eIF2a, and MyHC. (**c**) The statistical analyses results of the Western blot of the phosphorylation level of mTOR, S6, 4E-BP1, eIF2a, and MyHC for (**b**). Data are presented as mean ± SEM. *means *P* < 0.05 compared with the control. β-actin served as a housekeeping gene control.

**Figure 4:** mTOR signaling pathway mediated AKG-induced protein synthesis in C2C12 myotubes. (**a**) C2C12 myotubes were treated with 2 mM AKG for 1, 2, and 4 h. The expression levels of phosphorylation of mTOR, S6K, S6, 4E-BP1, eIF2a, and eIF4E were detected by Western blot. (**b**) C2C12 cells were cultured for 6 d in a differentiation medium. mTOR inhibitor rapamycin (1 μM) was used alone or co-treated with AKG (2 mM) for 48 h. Total protein levels. (**c**) The expression of puromycin determined by Western blot after C2C12 cells were co-treated with AKG and rapamycin. (**d**) The expression levels of phosphorylation of mTOR, S6, and 4E-BP1 detected by Western blot after C2C12 cells were co-treated with AKG and rapamycin. Data are presented as mean ± SEM. *means *P *< 0.05 compared with the control. β-actin served as a housekeeping gene control.

RETRACTED

**Figure 5:** Akt was required to enable AKG to activate mTOR signaling pathway and promote protein synthesis in C2C12 myotubes. (**a**) C2C12 myotubes were treated with AKG (2 mM) for 1, 2, and 4 h. The expression levels of MuRF1 and MAFbx and the phosphorylation of Akt FoxO1 and FoxO3a were then detected by Western blot. (**b**) C2C12 cells were cultured for 6 d in a differentiation medium. Akt inhibitor LY294002 (5 μM) was used alone or co-treated with AKG (2 mM) for 48 h. Total protein levels were detected. (**c**) The phosphorylation levels of Akt and FoxO1 by Western blot in C2C12 myotubes co-treated with AKG and LY294002. (**d**) The phosphorylation levels of mTOR, S6 and 4E-BP1 by Western blot in C2C12 myotubes co-treated with AKG and LY294002. Data are presented as mean ± SEM. *means *P *< 0.05 compared with the control. β-actin served as a housekeeping gene control.

**Figure 6:** Role of GPR91 in AKG-induced protein synthesis. C2C12 cells were transfected with vector or siGPR91. C2C12 cells were cultured for 6 d in a differentiation medium and then treated with AKG (2 mM) for 48 h. (**a**) The expression of GPR91 and GPR99 in C2C12 cells. (**b**) AKG up-regulated the mRNA expression of GPR91. (**c**) Total protein levels in C2C12 myotubes. (**d**) The phosphorylation levels of mTOR, S6, and 4E-BP1 measured by Western blot. (**e**) The mRNA expression of MuRF1 and MAFbx by qPCR. Data are presented as mean ± SEM. Different superscripts “a”/“b” represent significant differences between groups (*P *< 0.05), and *means *P *< 0.05 compared with the control. β-actin served as a housekeeping gene control. *n.d*. not detectable.

**Figure 7:** AKG regulated the protein synthesis of the skeletal muscle of mice. AKG (0.6 g/kg) and puromycin were co-injected for 3 h. Protein turnover associate protein expression was detected by Western blot. (**a**) The expression of puramycin was analyzed by Western blot. (**b**) The expression of MyHC and the phosphorylation levels of mTOR, S6, 4E-BP1, eIF4E, eIF2a in the gastrocnemius of mice. (**c**) The expression of Akt, MAFbx, and MuRF1. (**d**) The mRNA expression levels of protein turnover related genes were measured by qPCR. (**e**) The phosphorylation levels of Akt and mTOR 1 h after AKG injection detected by Western blot. Data are presented as mean ± SEM. *means *P* < 0.05 compared with the control. β-actin served as a housekeeping gene control.

RETRACTED

**Table 1:** PCR primer sequences and amplification parameters.

Gene	Primer sequence (5′-3′)	Product size (bp)	Tm (°C)
β-actin	S: 5′- GGTCATCACTATTGGCAACGAG -3′	142	57
	A: 5′- GAGGTCTTTACGGATGTCAACG -3′		
MAFbx	S: 5′- TCAGAGAGGCAGATTCGCAA -3′	154	59
	A: 5′- TCCAGGAGAGAATGTGGCAG -3′		
MuRF1	S: 5′- TTTGACACCCTCTACGCCAT -3′	203	59
	A: 5′- TTGGCACTTGAGAGGAAGGT -3′		
GPR91	S: 5′- TGTCACTGTGGTGTTTGGCTAC -3′	123	59
	A: 5′- GCATTTATCAGGATGGGAAGG -3′		
GPR99	S: 5′- CCTGCCATTGGTGATAGTGAC -3′	153	59
	A: 5′- GGGTGGAAGGGTAAGAAACAT -3′		
4E-BP1	S: 5′- TCAAGGCTGTGAGGTAGTCT -3′	186	59
	A: 5′- CTTGCATGGGAGGCTCATC -3'		

## References

[b1] FanzaniA., ConraadsV. M., PennaF.& MartinetW. Molecular and cellular mechanisms of skeletal muscle atrophy: an update. J Cachexia Sarcopenia Muscle 3, 163–179 (2012).2267396810.1007/s13539-012-0074-6PMC3424188

[b2] GordonB. S., KelleherA. R.& KimballS. R. Regulation of muscle protein synthesis and the effects of catabolic states. Int J Biochem Cell Biol 45, 2147–2157 (2013).2376996710.1016/j.biocel.2013.05.039PMC3759561

[b3] GlassD. J. Skeletal muscle hypertrophy and atrophy signaling pathways. Int J Biochem Cell Biol 37, 1974–1984 (2005).1608738810.1016/j.biocel.2005.04.018

[b4] WolfeR. R. Regulation of muscle protein by amino acids. Nutrition Week 2002 Meeting: SAN DIEGO, CALIFORNIA. AMER SOC NUTRITION-ASN. (FEB 27, 2002).10.1093/jn/131.10.3219S12368421

[b5] SuryawanA.& DavisT. A. Regulation of protein degradation pathways by amino acids and insulin in skeletal muscle of neonatal pigs. J Anim Sci Biotechnol 5, 8, doi: 10.1186/2049-1891-5-8 (2014).24438646PMC3901752

[b6] JeyapalanA. S. . Glucose stimulates protein synthesis in skeletal muscle of neonatal pigs through an AMPK- and mTOR-independent process. Am J Physiol Endocrinol Metab 293, E595–603 (2007).1755100210.1152/ajpendo.00121.2007

[b7] AthertonP. J.& SmithK. Muscle protein synthesis in response to nutrition and exercise. J Physiol 590, 1049–1057 (2012).2228991110.1113/jphysiol.2011.225003PMC3381813

[b8] SugdenP. H.& FullerS. J. Regulation of protein turnover in skeletal and cardiac muscle. Biochem J 273, 21–37 (1991).198958310.1042/bj2730021PMC1150210

[b9] DuranR. V. . Glutaminolysis activates Rag-mTORC1 signaling. Mol Cell 47, 349–358 (2012).2274952810.1016/j.molcel.2012.05.043

[b10] WhiteJ. P. . Testosterone regulation of Akt/mTORC1/FoxO3a signaling in skeletal muscle. Mol Cell Endocrinol 365, 174–186 (2013).2311677310.1016/j.mce.2012.10.019PMC3529800

[b11] GoodmanC. A. . The role of skeletal muscle mTOR in the regulation of mechanical load-induced growth. J Physiol 589, 5485–5501 (2011).2194684910.1113/jphysiol.2011.218255PMC3240886

RETRACTED

[b12] SchiaffinoS. e. a. Mechanisms regulating skeletal muscle growth and atrophy. FEBS J 280, 4294–4314 (2013).2351734810.1111/febs.12253

[b13] DeldicqueL. . Antagonistic effects of leucine and glutamine on the mTOR pathway in myogenic C2C12 cells. Amino Acids 35, 147–155 (2008).1797888810.1007/s00726-007-0607-z

[b14] ZhouJ. . FOXO3 induces FOXO1-dependent autophagy by activating the AKT1 signaling pathway. Autophagy 8, 1712–1723 (2012).2293178810.4161/auto.21830PMC3541283

[b15] CrosslandH., Constantin-TeodosiuD., GardinerS. M., ConstantinD.& GreenhaffP. L. A potential role for Akt/FOXO signalling in both protein loss and the impairment of muscle carbohydrate oxidation during sepsis in rodent skeletal muscle. J Physiol 586, 5589–5600 (2008).1881824110.1113/jphysiol.2008.160150PMC2655379

[b16] DuranR. V. . HIF-independent role of prolyl hydroxylases in the cellular response to amino acids. Oncogene 32, 4549–4556 (2013).2308575310.1038/onc.2012.465PMC3787797

[b17] HouY. . Alpha-Ketoglutarate and intestinal function. Front Biosci (Landmark Ed) 16, 1186–1196 (2011).2119622610.2741/3783

[b18] KristensenN. B., JungvidH., FernandezJ. A.& PierzynowskiS. G. Absorption and metabolism of alpha-ketoglutarate in growing pigs. Journal of Animal Physiology and Animal Nutrition 86, 239–245 (2002).1537991010.1046/j.1439-0396.2002.00380.x

[b19] JewellJ. L. . Metabolism. Differential regulation of mTORC1 by leucine and glutamine. Science 347, 194–198 (2015).2556790710.1126/science.1259472PMC4384888

[b20] YaoK. . Alpha-ketoglutarate inhibits glutamine degradation and enhances protein synthesis in intestinal porcine epithelial cells. Amino Acids 42, 2491–2500 (2012).2186116910.1007/s00726-011-1060-6

[b21] WeihaiH. . Citric acid cycle intermediates as ligands for orphan G-protein-coupled receptors. NATURE 429, 188–193 (2004).1514121310.1038/nature02488

[b22] DiehlJ. . Expression and localization of GPR91 and GPR99 in murine organs. Cell Tissue Res, doi: 10.1007/s00441-015-2318-1 (2015).26590824

[b23] WittenbergerT. . GPR99, a new G protein-coupled receptor with homology to a new subgroup of nucleotide receptors. Bmc Genomics 3, 17, doi: 10.1186/1471-2164-3-17 (2002).12098360PMC117779

[b24] WittenbergerT., SchallerH. C.& HellebrandS. An expressed sequence tag (EST) data mining strategy succeeding in the discovery of new G-protein coupled receptors. Journal of Molecular Biology 307, 799–813 (2001).1127370210.1006/jmbi.2001.4520

[b25] OnerJ., OnerH., SahinZ., DemirR.& UstunelI. Melatonin is as effective as testosterone in the prevention of soleus muscle atrophy induced by castration in rats. Anat Rec (Hoboken) 291, 448–455 (2008).1829337510.1002/ar.20659

RETRACTED

[b26] LaplanteM.& SabatiniD. M. mTOR signaling in growth control and disease. Cell 149, 274–293 (2012).2250079710.1016/j.cell.2012.03.017PMC3331679

[b27] FrumanD. A.& RommelC. PI3K and cancer: lessons, challenges and opportunities. Nat Rev Drug Discov 13, 140–156 (2014).2448131210.1038/nrd4204PMC3994981

[b28] SrikanthanP.& KarlamanglaA. S. Relative muscle mass is inversely associated with insulin resistance and prediabetes. Findings from the third National Health and Nutrition Examination Survey. J Clin Endocrinol Metab 96, 2898–2903 (2011).2177822410.1210/jc.2011-0435

[b29] YouJ. S., AndersonG. B., DooleyM. S.& HornbergerT. A. The role of mTOR signaling in the regulation of protein synthesis and muscle mass during immobilization in mice. Dis Model Mech 8, 1059–1069 (2015).2609212110.1242/dmm.019414PMC4582099

[b30] JufferP., BakkerA. D., Klein-NulendJ.& JaspersR. T. Mechanical loading by fluid shear stress of myotube glycocalyx stimulates growth factor expression and nitric oxide production. Cell Biochem Biophys 69, 411–419 (2014).2440267410.1007/s12013-013-9812-4

[b31] SnijdersT. . Protein Ingestion before Sleep Increases Muscle Mass and Strength Gains during Prolonged Resistance-Type Exercise Training in Healthy Young Men. J Nutr 145, 1178–1184 (2015).2592641510.3945/jn.114.208371

[b32] BentzingerC. F. . Differential response of skeletal muscles to mTORC1 signaling during atrophy and hypertrophy. Skelet Muscle 3, 6, doi: 10.1186/2044-5040-3-6 (2013).23497627PMC3622636

[b33] GoodmanC. A. . A phosphatidylinositol 3-kinase/protein kinase B-independent activation of mammalian target of rapamycin signaling is sufficient to induce skeletal muscle hypertrophy. Mol Biol Cell 21, 3258–3268 (2010).2066816210.1091/mbc.E10-05-0454PMC2938390

[b34] AretaJ. L., HawleyJ. A., YeJ. M., ChanM. H.& CoffeyV. G. Increasing leucine concentration stimulates mechanistic target of rapamycin signaling and cell growth in C2C12 skeletal muscle cells. Nutr Res 34, 1000–1007 (2014).2543902910.1016/j.nutres.2014.09.011

[b35] HeL.. The Physiological Basis and Nutritional Function of Alpha-ketoglutarate. Curr Protein Pept Sci 16, 576–581 (2015).2612277710.2174/1389203716666150630140157

[b36] PivaA., MorlacchiniM., PrandiniA., JungvidH.& PivaG., alpha-Ketoglutaric acid reduces nitrogen losses in rats fed nitrogen-free diet. 8th Symposium on Digestive Physiology in Pigs, Uppsala, Sweden. CABI Publishing. doi: 10.1079/9780851995175.0101 (June 20, 2000).

[b37] HammarqvistF., WernermanJ., von der DeckenA.& VinnarsE. Alpha-ketoglutarate preserves protein synthesis and free glutamine in skeletal muscle after surgery. Surgery 109, 28–36 (1991).1898624

RETRACTED

[b38] ProudC. G. mTOR-mediated regulation of translation factors by amino acids. Biochem Biophys Res Commun 313, 429–436 (2004).1468418010.1016/j.bbrc.2003.07.015

[b39] HaraK. . Regulation of eIF-4E BP1 phosphorylation by mTOR. J Biol Chem 272, 26457–26463 (1997).933422210.1074/jbc.272.42.26457

[b40] GaoP. . c-Myc suppression of miR-23a/b enhances mitochondrial glutaminase expression and glutamine metabolism. Nature 458, 762–765 (2009).1921902610.1038/nature07823PMC2729443

[b41] WalkerM. C.& van der DonkW. A. The many roles of glutamate in metabolism. J Ind Microbiol Biotechnol 43, 419–430 (2016).2632361310.1007/s10295-015-1665-yPMC4753154

[b42] HasebeM. . Glutamate in enteral nutrition: can glutamate replace glutamine in supplementation to enteral nutrition in burned rats? JPEN J Parenter Enteral Nutr 23, S78–82 (1999).1048390210.1177/014860719902300520

[b43] JaitovichA. . High CO_2_ levels cause skeletal muscle atrophy via AMP-activated kinase (AMPK), FoxO3a protein, and muscle-specific Ring finger protein 1 (MuRF1). J Biol Chem 290, 9183–9194 (2015).2569157110.1074/jbc.M114.625715PMC4423704

[b44] GlassD. J. PI3 kinase regulation of skeletal muscle hypertrophy and atrophy. Curr Top Microbiol Immunol 346, 267–278 (2010).2059331210.1007/82_2010_78

[b45] LiH. H. . Atrogin-1 inhibits Akt-dependent cardiac hypertrophy in mice via ubiquitin-dependent coactivation of Forkhead proteins. J Clin Invest 117, 3211–3223 (2007).1796577910.1172/JCI31757PMC2040316

[b46] BrooksN. E.& MyburghK. H. Skeletal muscle wasting with disuse atrophy is multi-dimensional: the response and interaction of myonuclei, satellite cells and signaling pathways. Front Physiol 5, 99, doi: 10.3389/fphys.2014.00099 (2014).24672488PMC3955994

[b47] Van GammerenD., DamrauerJ. S., JackmanR. W.& KandarianS. C. The IkappaB kinases IKKalpha and IKKbeta are necessary and sufficient for skeletal muscle atrophy. FASEB J 23, 362–370 (2009).1882702210.1096/fj.08-114249PMC2630783

[b48] FrostR. A.& LangC. H. Regulation of muscle growth by pathogen-associated molecules. J Anim Sci 86, E84–93 (2008).1819256010.2527/jas.2007-0483

[b49] YouJ. S., AndersonG. B., DooleyM. S.& HornbergerT. A. The role of mTOR signaling in the regulation of protein synthesis and muscle mass during immobilization. Dis Model Mech 8, 1059–1069 (2015).2609212110.1242/dmm.019414PMC4582099

[b50] ClavelS. . Regulation of the intracellular localization of Foxo3a by stress-activated protein kinase signaling pathways in skeletal muscle cells. Mol Cell Biol 30, 470–480 (2010).1991772110.1128/MCB.00666-09PMC2798458

[b51] BodineS. C. . Identification of ubiquitin ligases required for skeletal muscle atrophy. Science 294, 1704–1708 (2001).1167963310.1126/science.1065874

RETRACTED

[b52] SandriM. . Foxo transcription factors induce the atrophy-related ubiquitin ligase atrogin-1 and cause skeletal muscle atrophy. Cell 117, 399–412 (2004).1510949910.1016/s0092-8674(04)00400-3PMC3619734

[b53] ShinS. . ERK2 Mediates Metabolic Stress Response to Regulate Cell Fate. Mol Cell 59, 382–398 (2015).2619026110.1016/j.molcel.2015.06.020PMC4530034

[b54] WangY. . A “click” chemistry constructed affinity system for 2-oxoglutaric acid receptors and binding proteins. Org Biomol Chem 12, 6470–6475 (2014).2501927710.1039/c4ob01005a

[b55] LuC. Y. . Aberrant DNA methylation profile and frequent methylation of KLK10 and OXGR1 genes in hepatocellular carcinoma. Genes Chromosomes Cancer 48, 1057–1068 (2009).1976060810.1002/gcc.20708

[b56] NathansD. Inhibition of Protein Synthesis by Puromycin. Fed Proc 23, 984–989 (1964).14209831

[b57] HaggA. . Using AAV vectors expressing the beta2-adrenoceptor or associated Galpha proteins to modulate skeletal muscle mass and muscle fibre size. Sci Rep 6, 23042, doi: 10.1038/srep23042 (2016).26972746PMC4789796

